# LRSAM1 E3 Ubiquitin Ligase Promotes Choriocarcinoma Progression and Metastasis via p53/p21 Signaling Impediment

**DOI:** 10.1155/2022/1926605

**Published:** 2022-08-31

**Authors:** Qiumin Li, Ying Wang, Feifei Liu, Haili Wang, Yangyang Fan

**Affiliations:** Department of Obstetrics, Shaanxi Provincial People's Hospital, China

## Abstract

**Objective:**

The E3 ubiquitin ligase LRSAM1 (LRSAM1) was involved in many cancers, but whether it exerts anti- or protumor efficacies on choriocarcinoma cellular structures remains unknown. We wanted to explore the efficacies of aberrant LRSAM1 expression on human choriocarcinoma cellular structures and the underlying mechanisms.

**Methods:**

LRSAM1 mRNA expressions in choriocarcinoma lines of cells JEG-3 and JAR cellular structures, as well as HTR8/sev8 human trophoblastic cell line cellular structures, were assessed using assay analysis of quantitative real-time polymerase chain reactions. We compared cell proliferation, migratory flow, invasive force, adhesion, and apoptotic process between cellular structures infected with si-LRSAM1 plasmids versus negative controls using CCK-8, clone formation, Transwell, adhesion, and flow cytometry assays. Protein expressions of LRSAM1, E-cadherin, and N-cadherin (indicators of epithelial-mesenchymal transformation) and p53/p21 pathway components were quantitated using a Western blot assay. The morphology of tumor lesions was observed in xenografted nude mice using immunohistochemistry (IHC) analyses.

**Results:**

LRSAM1 was markedly overexpressed within JEG-3 and JAR choriocarcinoma cellular structures compared to HTR8/sev8 trophoblast cellular structures. Compared to si-NC, LRSAM1 knockdown robustly restricted cell proliferating, migratory flow, invasive force, and adhesion and fueled apoptotic cell process in JEG-3 as well as JAR cellular structures and suppressed tumor growth, as evidenced by the reduction in tumor volume and weight in naked mice inoculated with transfected cellular structures. Compared to si-negative control (si-NC), si-LRSAM1 significantly decreased Ki67 (a proliferating indicator) and N-cadherin expressions but reduced E-cadherin expression in JEG-3 and JAR cellular structures. Blocking the p53/p21 pathway by pifithrin-a (a p53 restrictor) successfully reversed the anti-inhibitory effect of LRSAM1 depletion, resulting in enhanced proliferating and metastasis in JEG-3 and JAR cellular structures.

**Conclusion:**

LRSAM1 exerts tumorigenic roles in choriocarcinoma. Via the activating of the p53/p21 pathway of signaling and impediment of choriocarcinoma cell proliferating, migratory flow, and invasive force, LRSAM1 knockdown slows the course of the disease. For choriocarcinoma diagnosis and treatment, it serves as a new therapeutic target.

## 1. Introduction

Choriocarcinoma is a very aggressive malignant trophoblastic tumor and the most prevalent epithelial tumor that primarily occurs in females. It originates from placental chorionic villi, fetal trophoblastic tissues, or abnormally proliferated trophoblasts during pregnancy [1, 2], characterized by malignant growth, widespread metastasis, and abnormal invasive force to the lungs, brain, and liver. For far too long, no effective treatment has been reported [3–5], primarily attributed to a lack of complete knowledge of precise mechanisms responsible for tumorigenesis. However, this information will be insightful for future studies of choriocarcinoma occurrence and new drug development for choriocarcinoma.

Current findings reveal that the E3 ubiquitin ligase LRSAM1 initiates autophagosome formation to capture invading bacteria, which are subsequently ubiquitinated and degraded [6, 7]. LRSAM1 depletion may interfere with neuronal development and homeostasis since it causes peripheral nerve axon degeneration and enhances axonal sensitivity in mice with Charcot-Marie-Tooth disease [8]. LRSAM1 expression was considerably elevated in colorectal cancer patients, according to Piepoli et al. [9], suggesting that abnormal LRSAM1 expression may contribute to cancer development. LRSAM1 was reported to increase expressions of cell adhesion molecules and promote glycogen synthase kinase phosphorylation in PC12 cellular structures via activation of the Wnt signaling [10], which is a critical mechanism for neuronal development [11]. Weterman et al. demonstrated that LRSAM1 promoted brain and spinal cord development and tail formation in Drosophila melanogaster, and *LRSAM1* knockdown significantly disturbed those processes [12].

Most studies of LRSAM1 in tumors support its role as a tumor suppressor, but whether it exerts anti- or protumor efficacies on choriocarcinoma cellular structures remains unknown. In the current research, we assessed LRSAM1 expression in choriocarcinoma cellular structures and the possible impact of aberrant LRSAM1 expression on malignant behaviors and transition from epithelium to mesenchyme and the involvement of critical signaling *experimentally and experimentally*. Moreover, the efficacies of p53/p21 signaling upon the cancer progression have been demonstrated previously. We speculated that LRSAM1 facilitated choriocarcinoma progression via p53/p21 signaling activation.

## 2. Materials and Methods

### 2.1. Cell Culture and Lines of Cells

ATCC, Manassas, Virginia provided the choriocarcinoma lines of cells JEG-3 and JAR cellular structures for humans, as well as the trophoblast cell line HTR8/sev8 cellular structures for humans (negative controls). Cellular structures were cultivated at 37°C in a humidified atmosphere, including five% CO_2_ in a RPMI-1640 medium containing 10% fetal bovine serum (Life Technologies, US) (FBS, Gibco, US).

### 2.2. Cell Transfection

JEG-3 and JAR cellular structures (1 × 10^5^ cellular structures/well) were sown in 6 deep dishes and nurtured until confluence reached 60-70%. The si-LRSAM1 were transfected into JEG-3 and JAR cellular structures using Lipofectamine 2000 (Invitrogen, US) for subsequent analyses for the efficacies of aberrant LRSAM1 expression on malignant behaviors of choriocarcinoma cellular structures and relevant mechanisms. LRSAM1 was detected with U6 as the internal reference, and others were detected with GAPDH as the internal reference. To determine the effectiveness of the transfection, transfected cellular structures were submitted to an RT-qPCR experiment. The following double-stranded siRNA sequences against LRSAM1 were utilized, and they were created. Genechem Incorporation (Shanghai, China) undertakes the chemical production of this product: si-LRSAM1-1: 5′-GCAGAUGACAUUCUCGACAUCUCUATT-3′, si-LRSAM1-2: 5′-CCGGCUCAUCCAGAUGGCCUACGAATT-3′.

### 2.3. Quantitative Real-Time PCR (qRT-PCR) Analysis

Genomic DNA was excerpted from cell lysates via TRIzol reagent (Takara, Japan) and afterward downward transcribed to cDNA via a PrimeScript RT reagent set (Takara, Japan) (Takara, Japan). In a real-time PCR detection system, the qRT-PCR was conducted using a standard SYBR premix Ex Taq (Takara, Japan) (Takara, Japan). Utilizing a fluorescence quantitative PCR 7500 system (ABI, US) and a miRcute miRNA qPCR set (TIANGEN, China) (TIANGEN, China), miRNA expressions were quantitated and standardized to internal controls GAPDH and U6. The 2^-*ΔΔ*Ct^ technique was utilized to calculate the relative fold gene expressions. For accuracy, each sample was examined in three different ways.

### 2.4. Cell Vivacity Assay

Inside RPMI-1640 media, including 10% FBS, cellular structures were suspended. Inside plates with 96 wells, cellular structures concentrated at 10^3^/100 *μ*L were injected, cultivated for one hour, and then mixed with 10 *μ*L of CCK-8 solution (Dojindo, Kumamoto, Japan) for two hours of incubation. A Bio-EL340 automatic microplate reader was utilized to assess the density of optics at 450 nm (Tek Instruments, Hopkinton, US).

### 2.5. Clone Formation Assay

Colony formation analysis was conducted to compare cell proliferating in JEG-3 and JAR cellular structures transfected versus uninfected with si-LRSAM1 plasmids. RPMI-1640 medium including 10% FBS was utilized to sustain transfected cellular structures (1 × 10^5^ cellular structures/well) for fourteen days. On day 15, the medium was withdrawn, and colonies were set in 4% paraformaldehyde for 30 minutes. 30 minutes after being stained with crystal violet, the cells were collected and photographed under a microscopic examination.

### 2.6. Flow Cytometry (FACS) Analysis

After being cultivated in 12-well plates with 1 × 10^5^ cellular structures/well JEG-3 and JAR cellular structures per well for 24 hours in serum-free RPMI-1640 media, the cellular structures were shaken for 5 min at 150 g at a speed of g. then twice rinsed with precooled 1PBS. The cellular structures were then preserved in 70% ethanol (CEF 590056, Solarbio, Peking, China) for 15 minutes at 20 degrees, centrifugation at 150 g for 5 minutes, and washed twice with chilled 1PBS. To eliminate residual RNA, cellular structures were treated for 45 minutes at 37 degrees with 10 g/L DNase-free RNase A (Sigma, Saint Louis, US). After two washes with ice-cold 1PBS, the cellular structures were centrifuged at 150 g for 5 minutes and then treated with 1 mg/mL iodide (Sigma, Saint Louis, US) for 12 minutes at 4°C in the dark. This action was taken to remove any residual RNA. Olympus, Tokyo, Japan, used FACS analysis to evaluate the distribution of cellular structures at each phase of the cell cycle and to identify cell apoptosis using an Annexin-FITC/PI apoptosis Identification Kit (Beyotime, Nanjing, China). All FACS data were processed and analyzed with ModiFit software (Olympus, Tokyo, Japan).

### 2.7. Wound Healing Assay

Three copies of wound healing tests were carried out to evaluate cell migratory flow thoroughly. In 6 well plates, JEG-3 and JAR cellular structures were plated and grown using a complete medium. Then, we scratched the monolayer of cellular structures using a sterile 10 *μ*L pipette tip. Separated cellular structures were then rinsed three times in a serum-free solution. They were cultured for a further 24 hours. Wounded areas were observed and photographed using inverted microscopy (Leica, Wetzlar, Germany) for macroscopic healing evaluation.

### 2.8. Transwell Assays

We utilized a Transwell test to investigate the potential for invasive cell force. Serum-free RPMI-1640 media was utilized to suspend JEG-3 and JAR cellular structures. The top chamber of a 24-well Transwell dish (CU3409301, 8 *μ*L pore diameter, Corning, US) was seeded with 100 *μ*L of cellular solution. Part of the cellular structures infiltrated the Matrigel membrane (BD Biosciences) after 48 hours of incubation and connected to the bottom membrane. The littler compartment was supplied with 500 *μ*L of DMEM to which 10% FBS had been added. After 15 minutes of fixation with 4% paraformaldehyde, the Transwell chambers were stained with 0.1% crystal violet at room temperature for 30 minutes. The residual cellular formations in the upper chambers were subsequently eliminated using a cotton swab. The stained cellular structures were examined and counted under a microscope in five fields after three PBS washes.

### 2.9. Matrigel Adhesion Assay

For the Matrigel adhesion assay, 1 × 10^5^ JEG-3 and JAR cellular structures were seeded on 24-well dishes coated in advance with 0.04 *μ*g/*μ*L Matrigel blended in FBS-free media and cultivated throughout the night to 90-percentage confluence. Cellular structures were washed in a medium before the assay to enable cell attachment in the absence of whole serum. Three PBS washes were performed on nonadherent cellular structures. Overexpressed JEG-3 and JAR cellular structures were adhered to Matrigel-coated wells, fixed with 4% paraformaldehyde, stained with 1% UV light, and examined for viability using optical microscopy.

### 2.10. Western Blot Assessment

After extracting total protein lysates using RIPA solution (Beyotime, China), the total protein concentration was measured using a BCA protein assay kit (Beyotime, China). Each lane was loaded with 30 *μ*g of protein content, separated on 6%, 8%, or 10% SDS-PAGE gels, and transferred to PVDF membranes (Millipore, US). The membranes were treated overnight at four degrees Celsius with antibody (BAT100493, 1 : 1000, Abcam, US), rinsed three times in PBST, and then left at room temperature for two hours while being treated with the matching secondary antibodies after being incarcerated in 5% skim milk/PBS-Tween (PBST) for 2 hours. The software was utilized to quantify the protein bands after they were seen using ECL (Tanon, Shanghai, China).

### 2.11. Bioinformatics Analysis

The Human Protein Atlas (https://www.proteinatlas.org/) was utilized to download gene expression data for choriocarcinoma patients. LRSAM1 mRNA expression patterns across various tumors were analyzed.

### 2.12. Choriocarcinoma Xenografts In Vivo

Mice were acquired from Beijing Weitong Lihua Biological Company when they were 6 to 7 weeks with a weight of 20–22 grams. SiLRSAM1-transfected JEG-3 and JAR cellular structures (1 × 10^6^) were occurred by subcutaneously inoculating into the right flank to establish human choriocarcinoma xenografts. Mice inoculated with si-NC-transfected cellular structures were utilized as negative controls. On day 28, cervical dislocation was utilized to end the lives of every mouse after regular monitoring. Tumor volume was measured every five days, tumor lesions were immediately collected and weighed, and the following calculations were made: (length × width^2^)/2 is the tumor volume in millimeters (mm^3^). For each mouse, a lesion was bisected for histomorphological.

### 2.13. Discoloration with Hematoxylin and Eosin (H&E)

For H&E discoloration, tumor lesions were embedded in paraffin and fixed in 4% paraformaldehyde. The lesions were sliced into 4 *μ*m thickness sections using a microtome. Sections were deparaffinized and then H&E stained., as described previously [13]. At least three sections of a lesion were selected for histopathological analysis using a microscope.

### 2.14. Immunohistochemistry (IHC) Assay

The deparaffinized slices were dried and treated with H_2_O_2_, and a graded ethanol series was used to dehydrate. After incarceration with bovine serum and being soaked in 5% skim milk/PBS, they were treated through the night with monoclonal antibodies against Ki67, E-cadherin, and vimentin (CEA400492, 1 in 1000 dilutions). After three items of washing, they were incubated with the secondary antibody (1 in 500) and horseradish peroxidase- (HRP-) conjugated streptavidin. HRP activity was determined using a 3,3′-diaminobenzidine (DAB) substrate kit. Hematoxylin was utilized as a counterstain, and a light microscope was utilized to see the sections (Olympus Incorporation, Tokyo, Japan).

### 2.15. Statistical Analysis

All results were represented by the mean and median from three independent experiments. As required, unpaired Student *t*-tests or single-way ANOVA were utilized to find differences in categories. To conduct the statistical analysis, we employed GraphPad Prism 7 and SPSS version 13.0 (SPSS, Chicago, IL, US) (GraphPad Inc., San Diego, CA, US). The criterion for statistical validity was a *P* value less than 0.05.

## 3. Results

### 3.1. LRSAM1 Expressions Are Upregulated and LRSAM1 Knockdown Inhibits Cell Proliferation in Choriocarcinoma

We queried human LRSAM1 expression in common human malignant tumors from HPA (https://www.proteinatlas.org/) (Figure 1(a)) to analyze and compare LRSAM1 expression patterns between the choriocarcinoma cell line JEG-3 and JAR and the trophoblast cell line HTR8/sev8. LRSAM1 abundance in JEG-3 and JAR cellular structures was notably higher than in HTR8/sev8 (Figure 1(b)). This finding implied that LRSAM1 might be a vital bioindicator in choriocarcinoma progression.

We found that Si-LRSAM1-1 had a better inhibitory effect than Si-LRSAM1-2, so Si-LRSAM1-1 was used later. Si-LRSAM1 was transfected into JEG-3 and JAR cellular structures to inquire more about the roles of LRSAM1 in choriocarcinoma cell proliferating, and successful LRSAM1 knockdown was observed, as evidenced by highly downregulated *LRSAM1* mRNA expressions in RT-qPCR analysis (Figure 1(c)). Compared to si-NC, LRSAM1 knockdown reduced cell vivacity and proliferated in JEG-3 and JAR cellular structures (Figures 1(d) and 1(e)). To rule out the possibility of decreased cell vivacity induced by cell cycle arrest, we assessed cell distribution at each cell cycle phase and found that G1 arrest was only observed in the si-LRSAM1 group (Figure 1(f)). Western blot analysis further supported this discovery, showing decreased Cyclin D1 and Ki-67 expressions following LRSAM1 knockdown (Figure 1(g)).

### 3.2. LRSAM1 Depletion Curbs Cell Migratory Flow, Invasive Force, and Adhesion in Choriocarcinoma Cellular Structures

We assessed malignant behaviors of choriocarcinoma cellular structures to understand the roles of aberrant LRSAM1 expression in tumor development. Compared to si-NC, LRSAM1 knockdown sharply suppressed cell migratory flow (Figures 2(a) and 2(b)) and invasive force (Figure 2(c)) in JEG-3 and JAR cellular structures compared to si-NC. The expression levels of matrix metalloproteinase 2 (*MMP2*) and *MMP9* genes fell sharply in si-LRSAM1-transfected cellular structures (Figure 2(d)). LRSAM1 depletion has an anti-inhibitory effect on the choriocarcinoma cell migratory flow, invasive force, and adhesion.

### 3.3. LRSAM1 Knockdown Accelerates the Apoptotic Process and Inhibits EMT in Choriocarcinoma Cellular Structures

Restricted cell proliferating, migratory flow, and adhesion can be explained by the apoptotic process and EMT. Therefore, we explored the underlying roles of LRSAM1 in these abnormal cell behaviors using FACS analysis, see Figure 3(a). JEG-3 and JAR cellular structures infected with si-LRSAM1 had a greater rate of cell apoptotic process. The upregulation of proapoptotic Bax, cleaved-caspase 3, and cleaved-caspase 9 protein contents and impediment of antiapoptotic Bcl-2 expression in transfected cellular structures further supported an apoptotic effect of si-LRSAM1 (Figure 3(b)). EMT is a process by which epithelial cellular structures acquire the features of mesenchymal cellular structures in tumor progression. Protein expressions of the EMT indicators, E-cadherin, and N-cadherin were evaluated.  Figure 3(c) shows increased E-cadherin expression and reduced N-cadherin expression were observed in the si-LRSAM1 group.

### 3.4. LRSAM1 Knockdown Inhibits Tumorigenesis of Choriocarcinoma Xenografts in Nude Mice

The JEG-3 and JAR cellular structures above were further validated in choriocarcinoma xenografts in nude mice. Compared to si-NC, si-LRSAM1 significantly hindered tumor growth (Figures 4(a) and 4(b)), with reduced tumor weight and volume (Figure 4(c)). In the histological and IHC analysis of tumor sections, more Ki67- and N-cadherin-positive and fewer E-cadherin-positive cellular structures were detected in the si-LRSAM1 group versus si-NC (Figures 4(d)–4(f)). All these findings supported the antitumorigenic activity of LRSAM1 knockdown.

### 3.5. LRSAM1 Knockdown Inhibits Choriocarcinoma Cell Proliferating and Metastasis via Activation of the p53/p21 Pathway

We also detected expressions of p53/p21 pathway components to explore the potential mechanisms behind extensive impediment of malignant behaviors of choriocarcinoma cellular structures following LRSAM1 knockdown. The p53 inhibitor, pifithrin-a (PFT, 100 nM), was administered in transfected cellular structures. Compared to si-NC, LRSAM1 knockdown significantly boosted *TP53* and *CDKN1A* mRNA expression levels, which were reversed in the si-LRSAM1+PFT group (Figure 5(a)). Likewise, PFT treatment robustly suppressed p21 protein expression and p53 phosphorylation compared to the highest levels in si-LRSAM1-transfected cellular structures (Figure 5(b)). In addition, previous impediments of cell proliferating, migratory flow, invasive force, and adhesion in transfected JEG-3 and JAR cellular structures were partly restored after PFT treatment compared to untreated cellular structures (Figures 5(c)–5(f)). These findings indicate that LRSAM1 knockdown inhibits malignant cell behaviors of choriocarcinoma cellular structures via p53/p21 signaling activation.

## 4. Discussion

For far too long, despite advancements in diagnostics and therapeutic strategies for choriocarcinoma treatment, the survival of choriocarcinoma patients has not yet improved. The proposal for more effective bioindicators for early prediction or screening is still essential for a better prognosis for patients. In the present study, we reported LRSAM1 upregulation in choriocarcinoma and remarkable antitumorigenic efficacies of LRSAM1 knockdown on choriocarcinoma cellular structures and xenografts in nude mice, including impediment of cell proliferating, migratory flow, invasive force, and adhesion and enhanced apoptotic process. These efficacies of si-LRSAM1 are triggered via activation of p53/p21 signaling.

Cell migratory flow, invasive force, and metastasis in tumor cellular structures can be explained by cell motility, which is determined by the dynamic cytoskeleton in response to stimuli [14]. Tumor invasive force is an early signal of metastasis, and a bioindicator enabling early prediction of invasive tumor force is the priority. Wang et al. reported that RKIP overexpression suppressed colorectal cancer cell metastasis, and RKIP knockdown facilitated metastasis experimentally [15]. Engeholm et al. and Tang et al. found that LRSAM1 mutations were associated with neurological disorders including Charcot-Marie-Tooth and Huntington's diseases [16, 17]. Our study reported LRSAM1 knockdown for the extensive impediment of cell motility of choriocarcinoma. Future studies of the efficacy of si-LRSAM1 in predicting migratory flow and invasiveness in choriocarcinoma cellular structures are expected.

A set of modulators and cell signaling mediate the apoptotic process or the process of programmed cell death. The Bcl-2 family, which consists of pro- and antiapoptotic molecules like Bcl-2, is a vital apoptotic process regulator (e.g., Bax). Alterations in the levels of anti- and proapoptotic protein contents influence the apoptotic process [18]. In the present study, we found that LRSAM1 knockdown suppressed proapoptotic protein contents and boosted Bcl-2 expression, fully exerting an apoptotic effect on choriocarcinoma cellular structures.

EMT is a crucial first step for tumor cellular structures to develop the ability to spread or invade [19, 20]. EMT is a form of evolution where cellular structures lose their epithelial features and gain mesenchymal features. Several bioindicators have been reported to have strong associations with EMT. According to Zhang et al., GRIM-19 prevented the invasive force of colorectal cancer cellular structures and utilized EMT by deactivating the STAT3/HIF-1*α* signaling [21]. It has been demonstrated that REC8 reduces EGR1 expression to prevent gastric cancer cellular structures from undergoing EMT [22]. The epithelial bioindicators are crucial for tumor spread include E-cadherin and vimentin [23–26]. In the present study, our findings demonstrated that LRSAM1 knockdown effectively reversed EMT, featuring a lower expression of the mesenchymal indicator N-cadherin and a higher expression of the epithelial indicator E-cadherin.

Current evidence supports that *TP53* (the tumor suppressor) gene therapy aids in the success of conventional chemotherapy, most of which leads to DNA damage, exerting persistent anti-tumor efficacies via p53-mediated apoptotic process and impediment of cell proliferating [27–30]. In this study, PFT (a p53 inhibitor) was administered to explore the potential roles of the p53/p21 signaling in si-LRSAM1's impediment of choriocarcinoma cell behaviors. The results showed that PFT treatment thwarted the transcriptional regulation of p21 via binding to p53, thus promoting cellular proliferating, migratory flow, and invasive force in choriocarcinoma.

In summary, LRSAM1 is extensively expressed in choriocarcinoma cellular structures and accelerates choriocarcinoma progression and metastasis via the p53/p21 signaling. LRSAM1 knockdown hinders choriocarcinoma progression, inhibiting choriocarcinoma cell proliferating, migratory flow, and invasive force and accelerating cell apoptotic process *experimentally and experimentally* via p53/p21 signaling activation. Thus, LRSAM1 may act as a prognostic bioindicator for choriocarcinoma.

Although our study confirmed that LRSAM1 might facilitate choriocarcinoma progression via p53/p21 signaling activation, our study still has some limitations and needs further improvement. We can supplement animal studies to further analyze the effects of LRSAM1 on choriocarcinoma in vivo. We will gradually improve around these aspects in the future.

## Figures and Tables

**Figure 1:** LRSAM1 expression is upregulated, and LRSAM1 knockdown inhibits cell proliferation in choriocarcinoma. (a) LRSAM1 overexpression is observed in choriocarcinoma patients from the Human Protein Atlas. (b) Significant LRSAM1 upregulation in JEG-3 and JAR choriocarcinoma cellular structures versus HTR8/sev8 cellular structures. (c) RT-qPCR assay reveals the successful knockdown of the *LRSAM1* gene. (d) The CCK-8 assay shows restricted cell vivacity in JEG-3 and JAR cellular structures versus HTR8/sev8 cellular structures. (e) Clone formation assay reveals hindered proliferating in JEG-3 and JAR cellular structures versus HTR8/sev8 cellular structures. (f) FACS analysis reveals G1 arrest that is only detectable in the si-LRSAM1 group. (g) Western blot shows lower expressions of cell cycle-related protein contents, Cyclin D1 and Ki-67, following LRSAM1 knockdown.

**Figure 2:** LRSAM1 depletion curbs cell migratory flow, invasive force, and adhesion in choriocarcinoma cellular structures. (a–c) The wound healing, Transwell migratory flow, and Matrigel adhesion assays reveal significant impediment of cell migratory flow and invasive force in si-LRSAM1-transfected JEG-3 and JAR cellular structures versus the si-NC group. (d) MMP-2 and MMP-9 protein expressions dropped markedly after LRSAM1 knockdown in JEG-3 and JAR cellular structures.

**Figure 3:** LRSAM1 knockdown accelerates apoptotic process and inhibits EMT in choriocarcinoma cellular structures. (a) FACS analysis shows enhanced cell apoptotic process. (b) Western blot reveals upregulation of proapoptotic Bax, cleaved-caspase 3, cleaved-caspase 9, and impediment of anti-apoptotic Bcl-2 in transfected cellular structures. (c) In transfected cellular structures, Western blot reveals a greater expression of E-cadherin and a decreased expression of N-cadherin.

**Figure 4:** LRSAM1 knockdown inhibits tumorigenesis of choriocarcinoma xenografts in nude mice. (a) Tumorigenesis and (b) tumor growth are examined in xenograft mice inoculated with si-LRSAM1-transfected JEG-3 and JAR cellular structures. (c) Reduced tumor weight and volume in xenograft mice.

**Figure 5:** LRSAM1 knockdown inhibits choriocarcinoma cell proliferation and metastasis via p53/p21 signaling activation. (a) The RT-qPCR assay shows significantly increased *P53* and *P21* mRNA expressions in the si-LRSAM1 group versus si-NC. (b) Western blot results of p21, p53, and p-p53 protein in the control, si-LRSAM1, and si-LRSAM1+PFT group, in JEG-3 and JAR cellular structures. (c) PFT treatment help restore cell proliferating in transfected cellular structures, as indicated by colon formation analysis. (d–f) Transwell migratory flow and Matrigel adhesion assays reveal that PFT treatment improves cell migratory flow, invasive force, and adhesion in transfected cellular structures versus untreated controls.

## Data Availability

The data used to support the findings of this study are available from the corresponding author upon request.

## References

[1] Sekiya Y., Yamamoto E., Niimi K. (2017). C-Rel promotes invasion of choriocarcinoma cells via PI3K/AKT signaling. *Oncology*.

[2] Shih I. M. (2007). Gestational trophoblastic neoplasia--pathogenesis and potential therapeutic targets. *The Lancet Oncology*.

[3] Traboulsi W., Sergent F., Boufettal H. (2017). Antagonism of EG-VEGF receptors as targeted therapy for choriocarcinoma progression in vitro and in vivo. *Clinical Cancer Research*.

[4] Zheng J., Lu J., Cheng M., Xu C. (2010). Lung metastasis of human choriocarcinoma in mice: establishment of experimental metastatic model and its biological characteristics. *Zhonghua Fu Chan Ke Za Zhi*.

[5] Mamelak A. N., Withers G. J., Wang X. (2002). Choriocarcinoma brain metastasis in a patient with viable intrauterine pregnancy: case report. *Journal of Neurosurgery*.

[6] Huett A., Heath R. J., Begun J. (2012). The LRR and RING domain protein LRSAM1 is an E3 ligase crucial for ubiquitin- dependent autophagy of intracellular _Salmonella_ typhimurium. *Cell Host & Microbe*.

[7] Ng A. C., Eisenberg J. M., Heath R. J. (2011). Human leucine-rich repeat proteins: a genome-wide bioinformatic categorization and functional analysis in innate immunity. *Proceedings of the National Academy of Sciences*.

[8] Bogdanik L. P., Sleigh J. N., Tian C. (2013). Loss of the E3 ubiquitin ligase LRSAM1 sensitizes peripheral axons to degeneration in a mouse model of Charcot-Marie-Tooth disease. *Disease Models & Mechanisms*.

[9] Piepoli A., Palmieri O., Maglietta R. (2012). The expression of leucine-rich repeat gene family members in colorectal cancer. *Experimental Biology and Medicine (Maywood, N.J.)*.

[10] Li B., Su Y., Ryder J., Yan L., Na S., Ni B. (2003). RIFLE: a novel ring zinc finger-leucine-rich repeat containing protein, regulates select cell adhesion molecules in PC12 cells. *Journal of Cellular Biochemistry*.

[11] Mulligan K. A., Cheyette B. N. (2012). Wnt signaling in vertebrate neural development and function. *Pharmacology*.

[12] Weterman M. A., Sorrentino V., Kasher P. R. (2012). A frameshift mutation in LRSAM1 is responsible for a dominant hereditary polyneuropathy. *Human Molecular Genetics*.

[13] Wang Y. Q., Jiang D. M., Hu S. S. (2019). SATB2-AS1 suppresses colorectal carcinoma aggressiveness by inhibiting SATB2-dependent Snail transcription and epithelial-mesenchymal transition. *Cancer Research*.

[14] Gimona M. (2009). Mechanics and dynamics of the cytoskeleton. *Cell Motility and the Cytoskeleton*.

[15] Wang Y., Wang L. Y., Feng F. (2015). Effect of Raf kinase inhibitor protein expression on malignant biological behavior and progression of colorectal cancer. *Oncology Reports*.

[16] Engeholm M., Sekler J., Schöndorf D. C. (2014). A novel mutation in LRSAM1 causes axonal Charcot-Marie-Tooth disease with dominant inheritance. *BMC Neurology*.

[17] Tang B., Seredenina T., Coppola G. (2011). Gene expression profiling of R6/2 transgenic mice with different CAG repeat lengths reveals genes associated with disease onset and progression in Huntington's disease. *Neurobiology of Disease*.

[18] Yin X. M., Oltvai Z. N., Korsmeyer S. J. (1994). BH1 and BH2 domains of Bcl-2 are required for inhibition of apoptosis and heterodimerization with Bax. *Nature*.

[19] Saitoh M. (2018). Involvement of partial EMT in cancer progression. *Journal of Biochemistry*.

[20] Cho A. A., Bonavida B. (2017). Targeting the overexpressed YY1 in cancer inhibits EMT and metastasis. *Critical Reviews in Oncogenesis*.

[21] Zhang J., Chu D., Kawamura T., Tanaka K., He S. (2019). GRIM‐19 repressed hypoxia‐induced invasion and EMT of colorectal cancer by repressing autophagy through inactivation of STAT3/HIF‐1*α* signaling axis. *Journal of Cellular Physiology*.

[22] Zhao J., Geng L., Duan G. (2018). REC8 inhibits EMT by downregulating EGR1 in gastric cancer cells. *Oncology Reports*.

[23] Antony J., Thiery J. P., Huang R. Y. (2019). Epithelial-to-mesenchymal transition: lessons from development, insights into cancer and the potential of EMT-subtype based therapeutic intervention. *Physical Biology*.

[24] Lei H., Gao Y., Xu X. (2017). LncRNA TUG1 influences papillary thyroid cancer cell proliferation, migration and EMT formation through targeting miR-145. *Acta Biochimica et Biophysica Sinica*.

[25] Wang L., Wei Z., Wu K. (2018). Long noncoding RNA B3GALT5-AS1 suppresses colon cancer liver metastasis via repressing microRNA-203. *Aging*.

[26] Liu C., Guan H., Wang Y. (2015). miR-195 inhibits EMT by targeting FGF2 in prostate cancer cells. *PLoS One*.

[27] Gao W., Shen Z., Shang L., Wang X. (2011). Upregulation of human autophagy-initiation kinase ULK1 by tumor suppressor p53 contributes to DNA-damage-induced cell death. *Cell Death and Differentiation*.

[28] Osawa T., Davies D., Hartley J. A. (2011). Mechanism of cell death resulting from DNA interstrand cross-linking in mammalian cells. *Cell Death & Disease*.

[29] Gatta R., Dolfini D., Mantovani R. (2011). NF-Y joins E2Fs, p53 and other stress transcription factors at the apoptosis table. *Cell Death & Disease*.

[30] Medema R. H., Macurek L. (2012). Checkpoint control and cancer. *Oncogene*.

